The article "Tuberculosis Disease Diagnosis Based on an Optimized Machine Learning Model" was published in 2022. Journal: J Healthc Eng.

# Tuberculosis Disease Diagnosis Based on an Optimized Machine Learning Model

**DOI:** 10.1155/2022/8950243

**Published:** 2022-03-21

**Authors:** Olfa Hrizi, Karim Gasmi, Ibtihel Ben Ltaifa, Hamoud Alshammari, Hanen Karamti, Moez Krichen, Lassaad Ben Ammar, Mahmood A. Mahmood

**Affiliations:** ^1^Department of Computer Science, College of Arts and Sciences at Tabarjal, Jouf University, Jouf, Saudi Arabia; ^2^STIH, Sorbonne Universite, Paris, France; ^3^Department of Information Systems, College of Computer and Information Sciences, Jouf University, Jouf, Saudi Arabia; ^4^Departement of Computer Sciences, College of Computer and Information Sciences, Princess Nourah Bint Abdulrahman University, P.O. Box 84428, Riyadh 11671, Saudi Arabia; ^5^Faculty of CSIT, Al-Baha University, Saudi Arabia & ReDCAD Laboratory, University of Sfax, Sfax, Tunisia; ^6^College of Sciences and Humanities, Prince Sattam Bin Abdulaziz University, Al-Kharj, Saudi Arabia

## Abstract

Computer science plays an important role in modern dynamic health systems. Given the collaborative nature of the diagnostic process, computer technology provides important services to healthcare professionals and organizations, as well as to patients and their families, researchers, and decision-makers. Thus, any innovations that improve the diagnostic process while maintaining quality and safety are crucial to the development of the healthcare field. Many diseases can be tentatively diagnosed during their initial stages. In this study, all developed techniques were applied to tuberculosis (TB). Thus, we propose an optimized machine learning-based model that extracts optimal texture features from TB-related images and selects the hyper-parameters of the classifiers. Increasing the accuracy rate and minimizing the number of characteristics extracted are our goals. In other words, this is a multitask optimization issue. A genetic algorithm (GA) is used to choose the best features, which are then fed into a support vector machine (SVM) classifier. Using the ImageCLEF 2020 data set, we conducted experiments using the proposed approach and achieved significantly higher accuracy and better outcomes in comparison with the state-of-the-art works. The obtained experimental results highlight the efficiency of modified SVM classifier compared with other standard ones.

## 1. Introduction

Tuberculosis (TB) is a highly contagious disease mainly affecting the lungs (called “pulmonary TB”). When it affects other organs, it is called “extrapulmonary TB.” It has rapidly spread all over the world and is currently considered one of the biggest threats to humanity. In 2015, the World Health Organization (WHO) estimated that TB caused over 1.8 million deaths worldwide [1, 2]. It is a clinical condition usually caused by a bacterium known as Mycobacterium tuberculosis [3]. Given that it affects multiple vital organs, it can be classified as a multisystem infectious disease. TB can also be classified as either “latent” or “active.” In 2018, WHO estimated that 25% of the world's population suffers from latent TB [4]. From this organization, TB disease can be categorized into different types such as skeletal TB that spreads to bones from lungs. It is rare. Also, miliary TB affected the lungs and bone marrow but can spread to other parts of the body such as the brain or heart. Liver TB is considered from rare TB forms. It accounts for less than 1% of all TB infections. All of these types occurred after the appearance of some clinical symptoms such as coughing, fever, weight loss, and night sweats. So, it can be life-threatening if not properly treated. Therefore, early detection and diagnosis are the most effective prevention method. Automatic TB diagnosis and classification techniques have been used in recent decades to improve the accuracy of disease recognition, thereby helping cardiologists make better decisions. Early techniques mainly used machine learning methods for automatic heartbeat classification, but required steps such as feature selection, feature extraction, and TB classification.

The article "Tuberculosis Disease Diagnosis Based on an Optimized Machine Learning Model" was published in 2022. Journal: J Healthc Eng.

Machine learning (ML) is a branch of artificial intelligence that develops mathematical models using training data. Its objective is to give a precise diagnosis that makes decisions without being manually programmed for specific tasks. Mitchell gives an old, but still valid, definition in [5]. ML is of great interest to researchers owing to its ability to answer fundamental scientific and technical questions, as well as to improve the highly practical computer software produced and used in many applications [6–10], such as the medical field.

Several studies indicate that image processing techniques have been applied to diverse areas of research, such as security, engineering science, medical diagnosis [11], and film. Computer algorithms are used in image processing to enhance, restore, filter, classify, compress, segment, or threshold, enabling researchers to draw conclusions based on points of interest [12, 13]. Medical imaging—i.e., the process of visually portraying the inside of the human body [14]—can be used for medical treatment and clinical analysis. It is not just a basic method of detection, but can also provide diagnoses for various diseases.

This work concerns the medical imaging research field, focusing on TB. Diverse images have been developed for use with medical image technology, such as magnetic resonance imaging (MRI), computerized tomography (CT) scans, and X-rays. These technologies are necessary for accurate diagnostic imaging tests and are important in choosing the ideal treatment plan. All of them can be intensively analyzed and processed [12]. This technique is called image processing and is one of the branches of computer science [15]. It performs operations on images to extract data according to specific criteria and a well-ordered sequence of steps [16]. A representative technique for this process is segmentation, which divides a given image into multiple segments (sets of pixels, also known as super-pixels). Segmentation is typically used to identify objects or other relevant information in digital images. There are many different methods or algorithms for image segmentation [17].

The article "Tuberculosis Disease Diagnosis Based on an Optimized Machine Learning Model" was published in 2022. Journal: J Healthc Eng.

Once image processing has been executed, the next step is the classification of the medical data. This stage was developed to overcome potential problems, with the objective of achieving promising results in the diagnosis of TB [18]. It is a system of categorizing all pixels within a digital image according to their characteristics, which are sorted into multiple sets of classes. Medical images are classified based on their extracted features. Input images may be classified as “normal” or “abnormal,” and “benign” or “malignant.” If each image is related to a unique one-class label or multi-label, the classification is single. If there are two class labels, the classification is binary; if there are more than two class labels, the classification is multiclass. Multiclass classification deals with a large number of labels [19], allowing each image to be tagged with more than one label. In this study, we use multiclass classification.

Feature extraction and representation is a crucial step in image processing, especially in the construction of any pattern classification. It consists of extracting the features that most accurately reflect the content of the images and assigning labels. During image classification, image features are extracted and numbered and then organized into classes. Some of the extracted features are irrelevant, redundant, or correlated, and sometimes, background noise leads to reduced efficiency and performance. Selecting the most meaningful features is a crucial step in classification. It is essential to remove insignificant features from the data set in order to guarantee more accurate diagnoses in medical applications. The performance of the classification model depends largely on the number of image features, which represent the input data set of the training model. However, there has been very little research on this problem. The extraction and selection of the most relevant features are still a challenge in the field of computer vision, particularly in image classification. Few works have classified TB using the K-nearest neighbor algorithm, a radial basis function (RBF) network, a multilayer perceptron (MLP) network, and a kernel regression to distinguish between bacilli and non-bacilli [20]. Support vector machine (SVM) is one of the most notable techniques [21, 22]. In this study, it is used in conjunction with a genetic algorithm to identify the smallest possible number of characteristics and to make the best possible distinctions between those features.

The article "Tuberculosis Disease Diagnosis Based on an Optimized Machine Learning Model" was published in 2022. Journal: J Healthc Eng.

In this study, we propose an improved SVM based on an optimization algorithm for automatic TB classification. To improve the performance of the SVM classifier, we propose new image feature extraction and selection techniques that improve feature representation. In particular, we analyze the efficacy of fusing image feature extraction and selection techniques. The main contributions of this study are as follows:

- To quickly solve the quadratic optimization problem, particularly the problem of hyper-parameters, we invented an improved SVM classifier that attempts to classify the data set by finding its optimal parameters (C and *γ*).

- To improve the performance of the SVM classifier, we propose two different techniques—feature extraction and feature selection—to obtain the most relevant features. In feature extraction, potential distinguishing features were extracted using wavelet transform, which provides the most suitable scale to represent texture classification. The wavelet function offers a wide range of choices, whereas other options, such as Gabor filters, are less suitable due to their lack of orthogonality. The main purpose of the feature selection technique is to select a subset of input variables using cutout features with no predictive information while constructing a classification model. A genetic algorithm is used to identify the smallest possible collection of characteristics, allowing for the best possible discrimination between the retrieved features.

- To highlight the performance of the SVM classifier, this study offers a comparison between different machine learning algorithms based on accuracy rate.

The rest of this study is organized as follows: Section 2 reviews related works on TB detection techniques; our materials and methods are described in Section 3; to conclude, Section 5 offers closing thoughts and a discussion of future work, while Section 4 describes the experimental assessment of our enhanced SVM classifier and compress the findings to those from other ML techniques.

The article "Tuberculosis Disease Diagnosis Based on an Optimized Machine Learning Model" was published in 2022. Journal: J Healthc Eng.

## 2. Background

This section provides a brief description of support vector machines (SVMs) and then discusses related works in the fields of classification and disease diagnosis.

### 2.1. Support Vector Machine

Classification is a technique that trains with a suitable classifier to classify a given input. For our purposes, and given that our input data sets were not augmented, an SVM classifier was the better choice for tuberculosis (TB) classification. SVM is a powerful supervised classifier. It was first introduced to the statistical theory field in 1982 by Vapnick [23]; then, other studies demonstrated its effectiveness in various applications, such as medical diagnosis [24, 25]. Nowadays, SVM is used with a computational model, which increases its accuracy while decreasing its complexity, but also requires an improved SVM classifier. Its main goal is to construct optimal separating hyperplanes in higher dimensions, referred to as decision planes, as shown in Figure 1. Along with the hyperplanes, SVM transformed the original training data into multidimensional space for the purposes of classification. The middle line in Figure 1 represents the maximum margin hyperplane, which separates the two classes at the maximum distance from the closest data point [26].

The separating hyperplane can be linear or nonlinear.

### 2.2. Linear Separation

A hyperplane separates the input patterns in a linear type, presented by (2):

(1) $$\begin{array}{c} w^{\tau }X+b=0, \end{array}$$

where *W*^*T*^ is an adjustable weight vector and *b* is the bias term. For each training example *x*_*i*_, we have the following:

(2) $$\begin{array}{c} Ef\left(x\right)\left\{\begin{array}{c} \geq 0\text{for}y_{i}=+1,\\ \leq 0\text{for}y_{i}=-1. \end{array}\right. \end{array}$$

If *y* = 1, the input example is normal. If *y* = -1, the input example is abnormal. Suppose that for two hyperplanes *H*_1_ : *W*′*X*_1_+*b*=0 and *H*_2_ : *W*′*X*_2_+*b*=0, the smallest perpendicular distance to the data point from the hyperplane is calculated as 2/‖*W*‖, and the best separation hyperplane is the one that maximizes the margin. The maximum margin hyperplane selection created by the SVM increases the accuracy of the classification and limits the number of misclassifications.

### 2.3. Nonlinear Separation

The linear SVM can be extended to a nonlinear classifier using a nonlinear operator *φ*(.) to determine the input pattern *x* in a higher-dimensional space H. The nonlinear SVM classifier so obtained is defined as follows: it is possible to convert the linear SVM into a nonlinear classifier by employing the nonlinear operator varphi(.) to identify the input pattern *x* in a higher-dimensional space H, as shown in Figure 1. The following is the definition of the nonlinear SVM classifier that was obtained:

(3) $$\begin{array}{c} f\left(x\right)=W^{T}\varphi \left(X\right)+b. \end{array}$$

The transformed data *φ*(*X*) show linearity, but in terms of the original data ⋮*x* ∈ *R*^*n*^, the classifier is nonlinear. To determine the parameters of decision function *f*(*x*), it must follow the minimization criteria:

(4) $$\begin{array}{c} \text{Min}J\left(W,\varepsilon \right)=\frac{1}{2}{\left\|W\right\|}^{2}+C\sum \varepsilon_{I}\text{Subjectto:}y_{i}\left(W^{T}\varphi \left(X\right)+b\right)\geq 1-\varepsilon_{i}. \end{array}$$

Following data preprocessing, a genetic algorithm (GA) selects a selection of features and extracts them using the spatial gray-level dependence method (SGLDM).

The article "Tuberculosis Disease Diagnosis Based on an Optimized Machine Learning Model" was published in 2022. Journal: J Healthc Eng.

There are several common kernel functions, given: Linear *x*_*i*_ · *x*_*i*_ Polynomial of degree: *d* : (*x*_*i*_ · *x*_*i*_+1)^*d*^ Radial basis function (RBF) which is expressed as: exp((−‖*x*_*i*_ − *x*_*j*_‖^2^)/2*ϑ*^2^)

### 2.4. Related Works

In this section, we rely on pure medical references to better explain TB, its location, its tendency to spread, its severity, and other data. This helps researchers to diagnose with greater precision and to use the right scientific and medical data in their studies.

In 2018, Kristen et al. [27] provided a systematic analysis of diverse bacterial strains that cause TB. It is also worth mentioning [5], in which the author concludes not only that TB is the multifaceted disease but also that there are many tests for its diagnosis. We also refer to studies in computer science, which use different techniques and algorithms to identify TB. We review below the main steps involved in a fully automatic TB detection system: digital image acquisition and preprocessing techniques, image segmentation methods, and feature extraction and classification.

### 2.5. Digital Image Acquisition and Preprocessing Techniques

In the literature, several studies have been presented for automatic TB detection, giving current researchers the ability to analyze the presence of TB bacteria automatically and quickly from a solid database [28]. An automatic TB detection system is used to automatically analyze the presence of TB bacteria quickly using different steps. The first step is image acquisition and preprocessing. Thus, before performing the image acquisition, an essential part of the automatic TB detection system called autofocusing has to be done [29] to save time and provide a better focused image. Several methods have been proposed for autofocusing [30, 31]. The performance of each method depends on different factors such as image characteristics, noise, and other specifics in the image.

The article "Tuberculosis Disease Diagnosis Based on an Optimized Machine Learning Model" was published in 2022. Journal: J Healthc Eng.

Before processing the acquired images, a preprocessing step must be accomplished for the images to enhance their quality. Several preprocessing methods have been proposed to improve the contrast and brightness of an image. Susanto et al. [32] developed an approach to identify lung TB. Their study applied image preprocessing methods to make identification faster. In [33], the authors published the first systematic review in which diverse models were proposed for the prediction of TB treatment outcomes.

When the data set is not uniform and lacks fine textural features, the first image processing task is to obtain uniformity throughout the data set and improve the quality of the images. This technique also aims to reduce image backgrounds. Le in [34] used a small window to scan the lung region for TB classification. Additionally, image processing techniques such as image enhancement, segmentation, and feature extraction have been used in [35] for TB diagnosis.

To obtain input data, Poornimadevi et al. [36] employed X-ray images; in 2017, Antony and Banu [37] added filtering to the same input database. Other works used a computed tomography (CT) scan for ImageCLEF, which organized a challenge based on CT image analyses of TB patients in 2017 [38].

Another frequently cited technique is machine learning (ML), which is used to model training data. The authors in [39] recently evaluated ML models for their efficacy in estimating TB prognosis. Other researchers detailed the ML mechanism, citing the survey in [40] in the development of their concepts and applications. The authors in the last work defined ML as “the union of forces between statistics and computer sciences” and “the basis for artificial intelligence.” In [41], the authors propose a feature selection model for brain tumor classification. In this study, we propose a model in two aspects, the first one for feature selection in the tuberculosis classification field and the second one for hyper-parameter selection. We aim to find the optimal SVM (C, *γ*) parameters to improve our classifier.

To study ML techniques such as logistic regression (LR) and linear discriminant analysis (LDA), we refer to [42] to identify causes, risk factors, and effective treatments.

Other recent researches such as [43, 44] adopted the ML algorithm for tuberculosis prediction.

### 2.6. Image Segmentation Methods

Image segmentation is one of the most crucial axes in medical image analysis. Its goal is to distinguish which objects caused a given disease within the tissue. Many TB-specific studies have proposed several segmentation algorithms such as thresholding methods, including K-means (KM) clustering, neural network-based approaches, and Bayesian segmentation [45, 46]. Several works proposed well-known thresholding algorithms to segment microscopic images, and other metaheuristic algorithms, such as KM, fuzzy c-means (FCM), fast marching (FM) thresholding, and the firefly algorithm (FA), were developed to solve bilevel microscopic image thresholding problems.

The article "Tuberculosis Disease Diagnosis Based on an Optimized Machine Learning Model" was published in 2022. Journal: J Healthc Eng.

Other studies used neural network (NN)-based approaches to detect TB bacilli. Priya and Srinivasan [47] used digital TB images for image-level and object-level classifications based on the multilayer perceptron (MLP) NN. TB detection has also been implemented using deep learning-based processes [48]. Hwang et al. [49] developed a modified AlexNet and used transfer learning.

### 2.7. Feature Extraction Methods

After segmentation, some impurities and unwanted data may remain in the images, necessitating feature extraction. Feature extraction is the reduction in image feature values to obtain better results and greater speed during the classification process. Thus, the feature extraction process plays an important role in the design of a good classification model.

Techniques based on Fourier transform (FT) [12] and wavelet transform (WT) [14, 15] have been developed in this regard. WT performs time-frequency analysis, while FT merely examines frequency. This makes it a useful tool for pattern detection and time-space-frequency analysis.

### 2.8. Classification Methods

Small artifacts and undesired areas remain in the image even after segmentation has been performed. Different classification approaches, such as Bayesian classifiers, support vector machines (SVM), probabilistic neural networks (PNNs), and KNN classifiers, are used to extract true bacilli from these segments. The techniques presented in [50, 51] used traditional classifiers—namely the Bayesian, NN, and random forest (RF) classifiers—which seem to be inefficient in classifying overlapping bacilli. Hooda et al. [52] proposed three standard architectures (AlexNet, GoogleNet, and ResNet) to create a custom data set for TB classification. Chithra and Jagatheeswari [53] drew comparisons between different classifiers to verify that their fractional crow search-based support vector neural network was highly accurate and performed better than others.

On the other hand, we cannot deny that some studies resulted in poorly labeled approaches to classifying TB. With these approaches, the exact locations or outline boundaries cannot be provided to the system, but an image label is added to identify a given chest X-ray (CXR) as “normal” or “abnormal.” These works are shown in [54, 55].

The article "Tuberculosis Disease Diagnosis Based on an Optimized Machine Learning Model" was published in 2022. Journal: J Healthc Eng.

Other strategies were designed to detect multiple TB manifestations using a supervised approach, as with Jaeger et al. [56], who described a technique to classify TB based on different shape and texture descriptors.

SVM is another important classifier that can be used to detect and count the number of TB bacteria. It is described in [57] as a state-of-the-art classifier in real-world pattern recognition applications. The current TB literature includes reviews comparing this classifier with more classical ones, where each comparison is based on some specific criterion, such as the outcome of each classifier.

In [21], SVM was compared with convolutional neural network (CNN) models. The experimental results showed that the best overall accuracy was 98.84%, obtained by an SVM-radial basis function (RBF) network model.

The authors in [58] proposed an automatic TB detection system that is based on the Gaussian fuzzy neural network (GFNN) classifier. The GFNN classifier combines the fuzzy classifier and the neural work with the Gaussian mixture model. It classifies the segments of the images into few bacilli, non-bacilli, and overlapping bacilli. The proposed GFNN model has achieved overall better performance in comparison with the various classical models, such as SVM, Bayesian regularization, Levenberg Marquardt, and fuzzy hyperbolic-based decision tree.

The authors in [59] proposed a hybrid classifier that combines the decision tree and the deep belief network along with the Gaussian model for infection-level identification in TB diagnosis. The classifier implements two-level classification techniques. At first-level classification, the images are categorized into three classes, such as few bacilli, non-bacilli, and overlapping bacilli. On the other hand, the second-level classification finds the number of bacilli by counting the bacilli and measuring the density ratio to determine the infection level. By showing a comparative analysis, the proposed Gaussian model has achieved overall better performance in comparison with that of existing conventional models, such as SVM, Bayesian regularization, Levenberg Marquardt, fuzzy hyperbolic-based decision tree, and GFNN.

One major challenge in TB screening is the development of a classification algorithm that guarantees higher accuracy, with a strong performance and sensitivity percentage to support doctors in making the right diagnosis.

## 3. Materials and Methods

In this section, we will introduce the materials we used and then describe the approaches we followed to achieve automatic tuberculosis (TB) classification.

### 3.1. Data Sets

Medical data collection is generally based on data volume, annotation, accuracy, and reusability. Each medical image can be defined by its data elements, metadata, and identifier. In this work, the data are provided as 3D computed tomography (CT) scans in compressed Neuroimaging Informatics Technology Initiative (NIfTI) files with the extension “.nii” from ImageCLEF campaign (https://www.imageclef.org/2020/medical/tuberculosis). After the files are decompressed, three sets of slices can be extracted, corresponding to the three dimensions of the 3D image XYZ (512 x 512 pixels). However, some experiments indicated that the slices of the Y dimension produced better results than that of *X* and *Z* dimensions; in fact, TB identification did not require every slice. Thus, we only have to keep those that are potentially informative. After selecting the Y dimension, the data set that we used contained 264 images. It is not a large database, but we chose it for the sake of a fully automated approach. In Figure 2, we give an example of a sample picture and the different types of TB-related findings.

The article "Tuberculosis Disease Diagnosis Based on an Optimized Machine Learning Model" was published in 2022. Journal: J Healthc Eng.

## 4. Methodology

A whole system must be followed during medical image processing. It contains many functions and other iterative methods to perform the optimization algorithm. Our proposed methodology for TB detection is shown in Figure 3. The input is the CT scan image of a human lung. This image is then preprocessed to improve its quality, and the output is given to the feature extraction block, which generates the input for the classifier.

This system comprises four main stages:

1. Input data preprocessing
2. Feature extraction
3. Feature selection
4. SVM hyper-parameter selection.

Each step will be detailed throughout the rest of this section.

### 4.1. Preprocessing: Feature Extraction Using Wavelet Transform

There are several multi-resolution approaches to feature extraction, most prominently Fourier transform (FT) and wavelet transform (WT). We worked with WT, which is a general mathematical tool for analyzing complex data sets and signal processing. WT's capabilities include time-scale signal analysis, signal decomposition, and signal compression. A major drawback of the FT method is that it delivers the same frequency resolution throughout the window function's duration. Moreover, it does not capture the time-evolving impacts of frequencies in nonstationary signals, whereas WT functions do so by providing a hierarchy of scales, starting with the coarsest scale in either stationary or nonstationary signals, respectively. Consequently, WT was deemed the most suitable tool for feature extraction due to its capability of displaying a picture at a variety of various resolutions. WT is often produced from the mother wavelet, and it is one of the most widely used instances of frequency-domain analysis and computation.

The article "Tuberculosis Disease Diagnosis Based on an Optimized Machine Learning Model" was published in 2022. Journal: J Healthc Eng.

For feature extraction, we used the spatial gray-level dependence method (SGLDM) developed by Haralick [60]. With this statistical technique, the geographical distribution of gray levels is estimated by computing the second-order conditional probability density *g* (i, *j*, d). An element at (i, j) of the SGLD matrix indicates the likelihood that two cells with differing resolutions, oriented away from the horizontal line, would have gray-level values I and *j*, respectively.

In Figure 4, WT image decomposition uses successive high-pass and low-pass filters.

22 features described in Table 1 were extracted by WT due to its multi-resolution capabilities.

### 4.2. Feature Selection via Genetic Algorithm

Those characteristics that are portrayed as actual numbers that exist in a high-dimensional space are not always meaningful or significant. Some of them are irrelevant, redundant, correlated, and occasionally noisy, making the learning models more likely to be overfit, complicated, and difficult to understand. As a result of these characteristics, data mining applications have low efficiency and poor performance (e.g., classification). The reduction in data dimensionality and the reduction in computational complexity are both required to choose robust features from unlabelled data to solve these difficulties.

Feature selection aims to select the most important one of the original features to avoid overfitting. To accomplish this task, we used a new technique based on a genetic algorithm (GA) for unsupervised feature selection.

GAs are stochastic search techniques, based on natural genetics, which provide robust search capabilities in complex spaces. A GA is an iterative process that solves an optimization problem [44]. Each solution is obtained by means of an encoding/decoding mechanism, which requires us to represent the solution as a chromosome. This is repeated conversely. To indicate the lack or existence of a feature, it is represented by zero or one at position *i*. GAs begin with a randomly generated population of chromosomes. A fitness function measures the solution's quality and efficacy. So, the fitness function in (1) treats the chromosome as input and outputs its fitness value. The next phase is to choose the fittest individuals to be future parents. Individuals can be used to create new populations by applying reproductive operators such as crossover and mutation.

(5) $$\begin{array}{c} \text{fitness}=W_{\text{acc}}\times \text{Accuracy}+W_{ft}\times \frac{1}{N}, \end{array}$$

where *W*_*a*_*cc* represents accuracy weight, *W*_*f*_*t* represents feature weight, and *N* represents the number of features selected.

The article "Tuberculosis Disease Diagnosis Based on an Optimized Machine Learning Model" was published in 2022. Journal: J Healthc Eng.

CT scans for tuberculosis (TB) can benefit from applying GAs to guarantee that the best feature sets are selected for analysis. Competition among feature transformation matrices is maintained. For each matrix in this population, transformed patterns are computed by multiplying the input patterns by the matrix to obtain a collection of chosen features, as illustrated in Figure 5. These features are then given to a classifier.

The GA system seeks to discover *m* optimal features from *n* extracted features to improve classifier performance. Finally, the GA's major purpose is to reduce the dimensionality of modified patterns while increasing classification accuracy.

### 4.3. SVM Parameter Selection

A large number of kernel functions are used to aid the support vector machine (SVM) in its pursuit of the best solution. The polynomial, sigmoid, and radial basis function (RBF) kernels are often employed. Unlike linear kernel functions, RBF is the most commonly used kernel function because it can effectively categorize multidimensional data. To get the best possible results, we used an RBF kernel function in our SVM. C and *γ*, two of the most important RBF parameters used with SVMs, had to be adjusted accordingly. In the example above, the parameter C represents the cost of the penalty. Because the value of this parameter has an influence on the partitioning results in the feature space, the value of this parameter has a substantially bigger impact on classification outcomes than the value of the other parameters.

The best classification accuracy rate may be determined by selecting suitable values for the upper and lower limits (search interval), as well as for the jumping interval, during the search process. In addition to the parameters C and *γ*, additional variables, such as the quality of the features data set, may have an impact on the classification accuracy rate, such as the number of false positives. Examples of this include the correlations between characteristics, which have an impact on the categorization outcome.

It is necessary to tweak C and *γ* when using the RBF kernel. It has been established that improper selection of the two parameters might result in over- or underfitting in the model. The suggested GA-based technique is intended to optimize C and *γ* for the SVM. This study employs the RBF kernel function for the SVM classifier to accomplish our suggested technique. Classification accuracy and the quantity of chosen characteristics were utilized to build a fitness function.

The proposed GA-SVM approach is described in greater detail below:

**Step 1 .**

The article "Tuberculosis Disease Diagnosis Based on an Optimized Machine Learning Model" was published in 2022. Journal: J Healthc Eng.

A binary string representation of the parameters and chromosomes that reflects the SVM parameters is created.

**Step 2 .**

The initial population of chromosomes is randomly generated, and then, the population is initialized.

**Step 3 .**

The parameters that were chosen (C and *γ*) are located.

**Step 4 .**

To get the trained optimal SVM, you will need to run your data through it with the new parameters. This model predicts the test sets.

**Step 5 .**

Fitness is assessed. To compute the k-fold cross-validation accuracy, the optimum chromosomes and optimal pair (C, gamma) are entered into an SVM classifier for each chromosome.

**Step 6 .**

The maximum number of generations N must be reached before the end of the game, or the fitness value of the preceding *M* generations must be lower than the current generation. There is no further iteration is possible if both conditions are satisfied.

## 5. Results and Discussion

All proposed techniques were implemented on computed tomography (CT) scans of tuberculosis (TB) patients. The input data set was divided into the training and testing sets. After the data set was collected, feature extraction was applied using the spatial gray-level dependence method (SGLDM) technique. In this section, the findings obtained through experimental studies are presented in two sections: (1) the findings obtained using hyper-parameter selection and (2) the findings obtained using feature selection.

Python was used to develop the model, which was tested using RTX 2060 Graphics Card and 16 GB of RAM.

### 5.1. Data Set and Evaluation Metrics

We used the ImageCLEF 2020 (https://www.imageclef.org/2020/medical/tuberculosis) data set, which is freely available on the Internet, to evaluate our enhanced machine learning model. In this study, we used multi-label classification. Three labels were assigned to each lung: “lung affected,” “presence of pleurisy,” and “presence of caverns.” The “left lung affected” and “right lung affected” labels marked the presence of any kind of tuberculosis (TB)-associated damage in the left and right lungs, respectively. Tables 2 and 3 detail the distribution of patients within each label.

In this study, we were most interested in accuracy, which is a metric for evaluating the overall efficacy of the classifier. The accuracy metric measures the probability that a diagnostic test was correctly performed (i.e., the proportion of correctly classified images). It can be evaluated using the following formula:

(6) $$\begin{array}{c} |\text{Acc}=\frac{\left(\text{TP}+\text{TN}\right)}{\left(\text{TP}+\text{TN}+\text{FP}+\text{FN}\right)}, \end{array}$$

where TP indicates that the model correctly predicted the positive class. FP indicates that the model incorrectly predicted the positive class. FN indicates that the model incorrectly predicted the negative class. TN indicates that the model correctly predicted the negative class. All of these values are defined in Table 4.

The article "Tuberculosis Disease Diagnosis Based on an Optimized Machine Learning Model" was published in 2022. Journal: J Healthc Eng.

Using the model described in this research, we conducted a series of experiments. Comparing the outcomes of various machine learning methods is also part of our research, for that we use Sklearn (https://scikit-learn.org/stable/) as Python package. scikit-learn (also known as Sklearn) is the most useable and stable machine learning toolkit available for Python. This package contains a range of efficient tools for machine learning and statistical modeling, such as classification and regression, clustering, and dimensionality reduction, all of which are accessible through a consistent interface in the Python programming language.

### 5.2. SVM Hyper-Parameter Selection

To improve the performance of the support vector machine (SVM), it is critical to first decide which parameters should be employed. To do so, we used an adaptive genetic algorithm (GA) to discover the ideal parameters. The primary purpose of the GA was to select the optimal parameters from a large number of alternative values to ensure the maximum possible accuracy throughout the training and testing stages. The parameters of the GA are presented in Table 5.

As per the discussion of kernel functions at the end of Section 3, the radial basis function (RBF) kernel is the most useful in terms of defining the optimal values of constants *γ* and C. Note that *γ* is the width of the kernel function and C is the error/trade-off parameter, which adjusts the significance of the separation error in the creation of the separation surface. The methodology proposed in this work was evaluated based on its accuracy.  Table 6 shows the variation in classification accuracy scores, which ranged from 0.64 to 0.97. All values were assessed using the validation data set.

Here, we present some of the many suggestions resulting from variations in the parameters selected by the GA to show the limits of the accuracy rates for each class. We note that the mean accuracy obtained by the SVM classifier reached its maximum values, as compared to the parameters individually chosen by the GA. As noted in the previous section, the SVM classifier was approved for this study due to the moderate size of the data set.

### 5.3. Comparison between SVM and Best-Known Machine Learning Models

In this section, we compare performance algorithms based on accuracy rate. The classifiers are as follows:

- “KNN,” K-neighbor classifier [61].

- “CART,” decision tree classifier [62].

- “NB,” Gaussian NB [63].

- “LDA,” linear discriminant analysis [64].

- “RF,” random forest classifier [65].

The article "Tuberculosis Disease Diagnosis Based on an Optimized Machine Learning Model" was published in 2022. Journal: J Healthc Eng.

In Table 7, we compared our SVM classifier with the supervised machine learning classifiers KNN, CART, NB, LDA, and RF. The experimental results show that our SVM classifier was more accurate than the other classification algorithms, while KNN and LDA performed better than CART and NB.

### 5.4. Feature Selection

Table 8 gives the range of selected features, as well as the accuracy score obtained in each range. Using the selection method, the optimal features were selected based on a GA and then used as input for the SVM classifier. The highest accuracy was obtained with the [3 : 12] range. By filtering the range of selected features, we minimized the number of extracted features, thereby accelerating the process of training.

As noted in the previous section, the SVM classifier was approved for this study due to the moderate size of the data set. Our modified SVM classifier, based on optimal parameters and feature-based selection methods, strongly improves classification accuracy. The optimal features used as input for our classifier were selected using a GA. The experimental results show that the GA was able to minimize the dimensionality of the transformed patterns while maximizing classification accuracy. It is very clear that our SVM classifier has achieved satisfactory results and attained a high classification accuracy rate. We can therefore note that our SVM classifier attempts to classify data sets by finding an optimal hyperplane and thus solves a quadratic optimization problem. In conclusion, our optimal SVM model significantly outperformed other models in classifying TB. The combination of optimal parameters and feature-based selection methods improved the performance of the GA in extracting robust and significant features. In general, the performance of machine learning algorithms is heavily dependent on the set of features to which they are applied.

## 6. Conclusion

In this study, we dealt with the problem of tuberculosis (TB) disease classification. Our main conclusions are as follows: the methodology discussed in this study highlights several techniques used in the field of medical image processing. Wavelet transform was used in conjunction with the spatial gray-level dependence method to extract features from the data set. These were then selected using an optimization genetic algorithm (GA) and were used as input for the support vector machine (SVM) classifier. To improve the performance of the SVM classifier, we used two new techniques based on our GA. For the first technique, we used an adaptive GA to determine the optimal parameters from a range of values in order to guarantee the highest possible accuracy during the training and testing phases. The second technique was used to select a small number of original features (i.e., the most one's features) to avoid overfitting and reduce the dimensional of the data. Finally, our experimental results show that our modified SVM classifier was more accurate than other classification algorithms in classifying TB. This study proves that the quality of extracted features has a direct impact on the effectiveness of image classification. Additionally, the proposed classification model can help doctors automatically diagnose TB because it possesses all of the qualities described in this study: accurate, robust, and easy to control. In future works, several improvements can be made. In particular, we are planning to address hybrid deep learning-based TB detection for improving the obtained results.

The article "Tuberculosis Disease Diagnosis Based on an Optimized Machine Learning Model" was published in 2022. Journal: J Healthc Eng.

## Figures and Tables

**Figure 1:** Separating hyperplane.

**Figure 2:** Slices of typical CT images with three types of TB-related findings (https://www.imageclef.org/2020/medical/tuberculosis).

**Figure 3:** Illustration of the proposed approach.

**Figure 4:** Block diagram of feature extraction by applying WT and SGLDM.

**Figure 5:** Genetic algorithm.

**Table 1:** Extracted features.

Features (mean/range)	
Frequency domain (32,33, 34)	Spatial domain (32,35)
Angular second moment	Correlation
Contrast	Variance
Inverse difference moment	Sum variance
Sum average	Difference variance
Entropy, sum entropy, difference entropy	Information measure of correlation I
Cluster prominence	Information measure of correlation II
Cluster shade	Maximal correlation coefficient
Dissimilarity	Correlation matrix
Homogeneity and inverse difference normalized	Maximum probability
Energy	

**Table 2:** Class distribution in tuberculosis data set.

Label	Number of occurrences	Test
Left lung affected	211	75
Right lung affected	233	99
Caverns left	66	3
Caverns right	79	5
Pleurisy left	7	28
Pleurisy right	14	46

**Table 3:** The percentage of train and test data for each label.

	Left lung affected	Right lung affected	Left lung pleurisy	Right lung pleurisy	Left lung caverns	Right lung caverns
Train	211 (75%)	233 (82%)	7 (2%)	14 (4%)	66 (23%)	79 (28%)
Test	75 (63%)	99 (83%)	3 (3%)	5 (4%)	28 (23%)	46 (38%)

**Table 4:** Truth table.

	Outcomes	Disease	
Test	+	TP	FP
	-	FN	TN

**Table 5:** GA parameters.

GA property	Value/method
Size of generation	100
Initial population size	30
Selection method	Tournament
Number of crossover points	1
Crossover probability	0.9
Mutation method	Uniform mutation
Mutation probability	0.05

The article "Tuberculosis Disease Diagnosis Based on an Optimized Machine Learning Model" was published in 2022. Journal: J Healthc Eng.

**Table 6:** Sample of binary classification results based on an adaptive genetic algorithm.

	Accuracy					
	Left lung affected	Right lung affected	Caverns left	Caverns right	Pleurisy left	Pleurisy right
*C* = 1, *γ* = 35	0.76	0.82	0.78	0.74	0.97	0.95
*C* = 20, *γ* = 35	0.68	0.75	0.64	0.64	0.95	0.93
*C* = 8, *γ* = 35	0.69	0.74	0.69	0.65	0.95	0.94
*C* = 1.5, *γ* = 20	0.75	0.81	0.76	0.73	0.97	0.95
*C* = 1.5, *γ* = 100	0.73	0.81	0.78	0.71	0.97	0.95

**Table 7:** Comparison between performance algorithms based on the rate of accuracy.

	SVM	KNN	CART	NB	LDA	RF
Left lung affected	0.77	0.72	0.63	0.46	0.72	0.70
Right lung affected	0.82	0.80	0.69	0.74	0.81	0.81
Caverns left	0.78	0.76	0.68	0.72	0.75	0.75
Caverns right	0.77	0.73	0.51	0.42	0.76	0.68
Pleurisy left	0.97	0.97	0.95	0.82	0.95	0.97
Pleurisy right	0.95	0.95	0.93	0.89	0.93	0.95
Mean accuracy	0.84	0.82	0.73	0.67	0.82	0.81

**Table 8:** Sample of selected feature results for the left and right lung affected category.

Range of selected features	Left lung	Left lung
[1 : 20]	0.75	0.79
[3 : 12]	0.78	0.83
[3 : 14]	0.77	0.82
[3 : 20]	0.77	0.81
[3 : 10]	0.75	0.8

## Data Availability

The Tuberculosis “TB 2020” data set used to support the findings of this study were supplied by the ImageCLEF campaign under license and so cannot be made freely available. Requests for access to these data should be made to https://www.imageclef.org/2020/medical/tuberculosis/; all the information necessary to have the database and the access authorization are mentioned in the following link: https://www.imageclef.org/2020/medical/tuberculosis/. The necessary codes for the machine learning models are mentioned in the following link: https://scikit-learn.org/stable/

## References

[1] World Health Organization (2015). *Global Tuberculosis Report 2015*.

[2] Yakobi A., Porterfield J. Z., Toman J. (2019). Hiv, tuberculosis, and otogenic intracranial sepsis: a devastating disease with a subtle presentation. *Otology & Neurotology*.

[3] World Health Organization (2021). Tuberculosis. http://www.who.int/es/news-room/fact-sheets/detail/tuberculosis.

[4] Iseman D. M. (2013). Tuberculosis: history. https://www.nationaljewish.org/conditions/tuberculosis-tb/history.

[5] Tom M. (1997). *Mitchell. Machine Learning*.

[6] Abu Al-Haija Q., Krichen M., Abu Elhaija W. (2022). Machine-learning-based darknet traffic detection system for iot applications. *Electronics*.

[7] Mian Qaisar S., Alyamani N., Waqar A., Krichen M. (2022). Machine learning with adaptive rate processing for power quality disturbances identification. *SN Computer Science*.

[8] Qaisar S., Mihoub A., Krichen M., Nisar H. (2021). Multirate processing with selective subbands and machine learning for efficient arrhythmia classification. *Sensors*.

The article "Tuberculosis Disease Diagnosis Based on an Optimized Machine Learning Model" was published in 2022. Journal: J Healthc Eng.

[9] Srinivasan S., Ravi V., Sowmya V, Krichen M., Noureddine D. B., Soman K. P. Deep convolutional neural network based image spam classification.

[10] Mihoub A., Snoun H., Krichen M., Bel Hadj Salah R., Kahia M. Predicting covid-19 spread level using socio-economic indicators and machine learning techniques.

[11] Gasmi K., Ltaifa I. B., Lejeune G., Alshammari H., Ammar L. B., Mahmood M. A. (2021). Optimal deep neural network-based model for answering visual medical question. *Cybernetics & Systems*.

[12] Walia N., Singh H., Kumar Tiwari S., Sharma A. (2015). A decision support system for tuberculosis diagnosability. *International Journal of Soft Computing*.

[13] Venu Madhavan M., Ngoc Hoang Thanh D., Khamparia A., Pande S., Malik R., Gupta D. (2021). Recognition and classification of pomegranate leaves diseases by image processing and machine learning techniques. *Computers, Materials & Continua*.

[14] Zhou Y. (2019). *Medical Imaging: Principles and Applications*.

[15] Kamble M. P. A., Anagire M. V. V., Chamtagoudar M. S. N. (2016). Cxr tuberculosis detection using matlab image processing. *International Research Journal of Engineering and Technology*.

[16] Gonzalez R. C., Woods R. E. (2008). *Digital Image Processing*.

[17] Wang L., Chen R., Wang S., Zeng N., Huang X., Liu C. (2019). Nested dilation network (ndn) for multi-task medical image segmentation. *IEEE Access*.

[18] Krizhevsky A., Sutskever I., Hinton G. E, Pereira F., Burges C. J. C., Bottou L., Weinberger K. Q. (2012). Imagenet classification with deep convolutional neural networks. *Advances in Neural Information Processing Systems*.

[19] Alazaidah R., Kabir Ahmad F. (2016). Trending challenges in multi label classification. *International Journal of Advanced Computer Science and Applications*.

[20] Osman M. K., Mashor M. Y., Jaafar H. (2012). Performance comparison of extreme learning machine algorithms for mycobacterium tuberculosis detection in tissue sections. *Journal of Medical Imaging and Health Informatics*.

[21] Hasan H., Shafri H. Z. M., Habshi M., Habshi M. A comparison between support vector machine (SVM) and convolutional neural network (CNN) models for hyperspectral image classification.

[22] Rubio F., Martínez-Gómez J., Julia Flores M., Puerta J. M. (2016). Comparison between bayesian network classifiers and svms for semantic localization. *Expert Systems with Applications*.

[23] Vapnik V. (2006). *Estimation of Dependences Based on Empirical Data*.

[24] Guyon I., Weston J., Barnhill S., Vapnik V. (2002). Gene selection for cancer classification using support vector machines. *Machine Learning*.

The article "Tuberculosis Disease Diagnosis Based on an Optimized Machine Learning Model" was published in 2022. Journal: J Healthc Eng.

[25] Zhang J., Liu Y. Cervical cancer detection using svm based feature screening.

[26] Morariu D., Lucian N. V., Tresp V. (2006). Feature selection methods for an improved svm classifier. *International Journal of Computer and Information Engineering*.

[27] Wiens K. E., Woyczynski L. P., Ledesma J. R. (2018). Global variation in bacterial strains that cause tuberculosis disease: a systematic review and meta-analysis. *BMC Medicine*.

[28] Panicker R. O., Soman B., Saini G., Rajan J. (2016). A review of automatic methods based on image processing techniques for tuberculosis detection from microscopic sputum smear images. *Journal of Medical Systems*.

[29] Russell M. J, Douglas T. S Evaluation of autofocus algorithms for tuberculosis microscopy.

[30] Fernandes Costa Filho C. F., Fernandes Costa M. G., Kimura Junior A. (2012). Autofocus functions for tuberculosis diagnosis with conventional sputum smear microscopy. *Current Microscopy Contributions to Advances in Science and Technology*.

[31] Pertuz S., Puig D., Garcia M. A. (2013). Analysis of focus measure operators for shape-from-focus. *Pattern Recognition*.

[32] Rohmah R. N., Susanto A., Soesanti I., Tjokronagoro M. Computer aided diagnosis for lung tuberculosis identification based on thoracic x-ray.

[33] Peetluk L. S., Moreira Ridolfi F., Rebeiro P. F., Liu D., Rolla V. C., Sterling T. R. (2021). Systematic review of prediction models for pulmonary tuberculosis treatment outcomes in adults. *BMJ Open*.

[34] Kim L. Automated detection of early lung cancer and tuberculosis based on x-ray image analysis.

[35] ullah M., Bari M., Ahmed A., Naveed S. (2019). Lungs cancer detection using digital image processing techniques: a review. *Mehran University Research Journal of Engineering and Technology*.

[36] Poornimadevi C. S., Sulochana H. Automatic detection of pulmonary tuberculosis using image processing techniques.

[37] Antony B. (2018). Lung tuberculosis detection using x-ray images. *International Journal of Applied Engineering Research*.

[38] Dicente Cid Y., Liauchuk V., Kovalev V., Müller H. (2017). *Overview of Imageclef 2017 Tuberculosis Task – Predicting Tuberculosis Type and Drug Resistances*.

[39] Ferreira Da Silva Barros M. H. L., Oliveira Alves G., Florêncio Souza L. M. (2021). Benchmarking machine learning models to assist in the prognosis of tuberculosis. *Informatics*.

[40] Behera R., Das K. (2017). A survey on machine learning: concept, algorithms and applications. *International Journal of Innovative Research in Computer and Communication Engineering*.

[41] Ahmed K., Gasmi K., Anouar Ben Messaoud M., Benamrane N., Mohamed A. (2010). A hybrid approach for automatic classification of brain mri using genetic algorithm and support vector machine. *Leonardo Journal of Sciences*.

The article "Tuberculosis Disease Diagnosis Based on an Optimized Machine Learning Model" was published in 2022. Journal: J Healthc Eng.

[42] Callahan A., Shah N. H. (2017). Machine learning in healthcare. *Key Advances in Clinical Informatics*.

[43] Faruk O., Ahmed E., Ahmed S. (2021). A novel and robust approach to detect tuberculosis using transfer learning. *Journal of healthcare engineering*.

[44] Ali M. H., Khan D. M., Jamal K., Ahmad Z., Manzoor S., Khan Z. (2021). Prediction of multidrug-resistant tuberculosis using machine learning algorithms in swat, Pakistan. *Journal of healthcare engineering*.

[45] Raof R. A. A., Yusoff Mashor M., Md Noor S. S. (2018). Segmentation of Tb Bacilli in Ziehl-Neelsen Sputum Slide Images Using K-Means Clustering Technique.

[46] Ayas S., Dogan H., Gedikli E., Ekinci M. (2018). A novel approach for bi-level segmentation of tuberculosis bacilli based on meta-heuristic algorithms. *Advances in Electrical and Computer Engineering*.

[47] Priya E., Srinivasan S. (2015). Separation of overlapping bacilli in microscopic digital tb images. *Biocybernetics and Biomedical Engineering*.

[48] Minaee S., Boykov Y., Porikli F., Plaza A., Kehtarnavaz N., Terzopoulos D. (2021). Image segmentation using deep learning: a survey. *IEEE Transactions on Pattern Analysis and Machine Intelligence*.

[49] Hwang S., Kim H.-E., Jeong J., Kim H.-J. A novel approach for tuberculosis screening based on deep convolutional neural networks.

[50] Priya E., Srinivasan S. (2016). Automated object and image level classification of tb images using support vector neural network classifier. *Biocybernetics and Biomedical Engineering*.

[51] Singh J., Tripathy A., Garg P., Kumar A. Lung tuberculosis detection using anti-aliased convolutional networks.

[52] Hooda R., Mittal A., Sofat S. (2019). Automated tb classification using ensemble of deep architectures. *Multimedia Tools and Applications*.

[53] Chithra R. S, Jagatheeswari P. (2018). Fractional crow search-based support vector neural network for patient classification and severity analysis of tuberculosis. *IET Image Processing*.

[54] Arzhaeva Y., Hogeweg L., Jong P., Viergever M., Ginneken B. (2009). Global and local multi-valued dissimilarity-based classification: application to computer-aided detection of tuberculosis. *Med Image Comput Comput Assist Interv*.

[55] Melendez J., Van Ginneken B., Maduskar P., Philipsen R. H. H. M., Ayles H., Sanchez C. I. (2016). On combining multiple-instance learning and active learning for computer-aided detection of tuberculosis. *IEEE Transactions on Medical Imaging*.

[56] Jaeger S., Karargyris A., Antani S., George T. Detecting tuberculosis in radiographs using combined lung masks.

The article "Tuberculosis Disease Diagnosis Based on an Optimized Machine Learning Model" was published in 2022. Journal: J Healthc Eng.

[57] Thiyagarajan M., Bharathi N. (2016). Lung cancer detection using fuzzy auto-seed cluster means morphological segmentation and svm classifier. *Journal of Medical Systems*.

[58] Mithra K. S., Sam Emmanuel W. R. (2021). Gfnn: Gaussian-fuzzy-neural network for diagnosis of tuberculosis using sputum smear microscopic images. *Journal of King Saud University - Computer and Information Sciences*.

[59] Mithra K. S., Sam Emmanuel W. R. (2021). Gaussian model based hybrid technique for infection level identification in tb diagnosis. *Journal of King Saud University - Computer and Information Sciences*.

[60] Haralick R. M., Shanmugam K., Dinstein I. H. (1973). Textural features for image classification. *IEEE Transactions on Systems, Man, and Cybernetics*.

[61] Aidos H., Fred A. k-nearest neighbor classification using dissimilarity increments. *Lecture Notes in Computer Science*.

[62] Swain P. H., Hauska H. (1977). The decision tree classifier: design and potential. *IEEE Transactions on Geoscience Electronics*.

[63] Xu S. (2018). Bayesian Naïve Bayes classifiers to text classification. *Journal of Information Science*.

[64] Dorfer M., Kelz R., Widmer G. (2016). Deep Linear Discriminant Analysis. https://arxiv.org/abs/1511.04707.

[65] Kam Ho T. Random decision forests.

